The article "Hydrogen bonds are a primary driving force for de novo protein folding" was retracted in 2018. Reasons: contaminated materials; errors in the data; errors in the results or conclusions.

# Hydrogen bonds are a primary driving force for *de novo* protein folding

**DOI:** 10.1107/S2059798317015303

**Published:** 2017-11-10

**Authors:** Schuyler Lee, Chao Wang, Haolin Liu, Jian Xiong, Renee Jiji, Xia Hong, Xiaoxue Yan, Zhangguo Chen, Michal Hammel, Yang Wang, Shaodong Dai, Jing Wang, Chengyu Jiang, Gongyi Zhang

**Affiliations:** a Department of Biomedical Research, National Jewish Health, Denver, CO 80206, USA; b Department of Immunology and Microbiology, School of Medicine, University of Colorado Denver, Aurora, CO 80206, USA; c Department of Chemistry, University of Missouri, Columbus, Mississippi, USA; d Physical Biosciences Division, Lawrence Berkeley National Laboratory, Berkeley, CA 94720, USA; e Department of Biochemistry and Molecular Biology, Peking Union Medical College, Beijing 100005, People’s Republic of China

**Keywords:** hydrogen bonds, *cis*/*trans*-proline, protein folding

## Abstract

The protein-folding mechanism remains a major puzzle in life science. Purified soluble activation-induced cytidine deaminase (AID) is one of the most difficult proteins to obtain. Starting from inclusion bodies containing a C-terminally truncated version of AID (residues 1–153; AID^153^), an optimized *in vitro* folding procedure was derived to obtain large amounts of AID^153^, which led to crystals with good quality and to final structural determination. Interestingly, it was found that the final refolding yield of the protein is proline residue-dependent. The difference in the distribution of *cis* and *trans* configurations of proline residues in the protein after complete denaturation is a major determining factor of the final yield. A point mutation of one of four proline residues to an asparagine led to a near-doubling of the yield of refolded protein after complete denaturation. It was concluded that the driving force behind protein folding could not overcome the *cis*-to-*trans* proline isomerization, or *vice versa*, during the protein-folding process. Furthermore, it was found that successful refolding of proteins optimally occurs at high pH values, which may mimic protein folding *in vivo*. It was found that high pH values could induce the polarization of peptide bonds, which may trigger the formation of protein secondary structures through hydrogen bonds. It is proposed that a hydrophobic environment coupled with negative charges is essential for protein folding. Combined with our earlier discoveries on protein-unfolding mechanisms, it is proposed that hydrogen bonds are a primary driving force for *de novo* protein folding.

## Abstract 2

The yield of protein refolding is reciprocal to the number of proline residues in the target protein. Hydrogen bonds are the primary driving force for *de novo* protein folding

The article "Hydrogen bonds are a primary driving force for de novo protein folding" was retracted in 2018. Reasons: contaminated materials; errors in the data; errors in the results or conclusions.

## 1. Introduction   

The capacity for the immune system to defend against the countless environmental pathogens results from the immense diversification (over 10^15^ types) of high-affinity immuno­globulins. The first mechanism which partakes in the generation of this diversification is the process of V(D)J recombination, which involves the antigen-independent generation of an enormous population of B cells consisting of individual cells expressing B-cell receptors (BCRs) with unique antigen-binding specificities (Cobb *et al.*, 2006 ▸; Harwood & Batista, 2008 ▸). In the presence of a foreign antigen, some fraction of this B-cell population that is capable of binding to the antigen will become activated and thus proliferate and differentiate, and undergo processes that (i) further enhance the binding affinity between the immunoglobulin of the activated B cell and the antigen, which is known as somatic hypermutation (SHM), and (ii) change the class of immuno­globulin to trigger an immune response that is best suited to counter the particular antigen, which is known as class-switch recombination (CSR) (Di Noia & Neuberger, 2007 ▸; Chaudhuri *et al.*, 2007 ▸). In 2000, the 24 kDa protein activation-induced cytidine deaminase (AID) was identified as a master regulator responsible for SHM and CSR (Muramatsu *et al.*, 2000 ▸; Revy *et al.*, 2000 ▸). AID is proposed to function by deaminating cytidine residues on single-stranded DNA (ssDNA), thus converting them to uridines. The resultant base-pair mismatch coopts the activities of normal cellular mismatch repair (MMR) or base-excision repair (BER) to convert the mismatch to mutational and/or double-strand break (DSB) outcomes (Di Noia & Neuberger, 2007 ▸). Ultimately, the overall activity of both SHM and CSR mediated by AID leads to the final affinity maturation and effector-function modification of immunoglobulin. Recent studies have revealed that various aberrant AID activities can lead to an autosomal recessive form of hyper-IgM syndrome, chronic lymphocytic leukemia (CLL) and follicular lymphoma (FL) (Revy *et al.*, 2000 ▸; Kasar *et al.*, 2015 ▸; Scherer *et al.*, 2016 ▸).

One of the major limitations in AID research is that a method for the purification of large quantities of recombinant wild-type AID is absent. Consequently, *in vitro* assays that require more than trace amounts of AID have yet to be performed. Furthermore, owing to this conundrum, a high-resolution structure of wild-type AID has yet to be solved. Notably, AID is one of 11 members of the apolipoprotein B mRNA-editing catalytic polypeptide-like (APOBEC) protein family (Salter *et al.*, 2016 ▸). The members of this protein family share a conserved zinc-dependent deaminase sequence motif, yet each member performs very distinct roles owing to variations in the length, composition and spatial location of conserved secondary-structural features. These distinguishing features among the APOBEC family members were elucidated through various structural studies that highlighted subtle and/or flagrant differences between family members (Salter *et al.*, 2016 ▸; King *et al.*, 2015 ▸, Prochnow *et al.*, 2007 ▸; Holden *et al.*, 2008 ▸). Although the structures of homologs, orthologs and a highly mutated version of AID exist, and provide valuable insight into corroborating the deamination mechanism of AID, a high-resolution structure of wild-type AID, which would provide valuable information that distinguishes AID from the rest of the APOBEC family members, has yet to be determined. Here, we report a twinned crystal structure of truncated wild-type AID^153^ at 2.0 Å resolution. High concentrations of the protein were obtained by solubilizing the inclusion bodies and performing an *in vitro* gradational refolding process. Given the successful outcome of refolding and crystallization of AID^153^, the protein was an ideal model system to investigate another major mystery in protein science: the effects of proline on protein folding.

The article "Hydrogen bonds are a primary driving force for de novo protein folding" was retracted in 2018. Reasons: contaminated materials; errors in the data; errors in the results or conclusions.

The effects of proline isomerization in the unfolding and refolding of proteins has been an open area of investigation since 1975 (Brandts *et al.*, 1975 ▸). Although the exact role of proline isomerization in this context has been controversial, the general consensus implicates proline isomerization as having an impact in the kinetics of protein unfolding and refolding (Brandts *et al.*, 1977 ▸). Specifically, mutating a particular proline residue in a given protein appears to significantly influence, either positively or negatively, the rate at which the protein converts from an unfolded state to a folded state (Roderer *et al.*, 2015 ▸; Osváth & Gruebele, 2003 ▸). We hypothesized that prolines in the incorrect configuration are trapped in non-native, yet thermodynamically favorable, conformations/aggregates and are unable to adopt the native conformation. From our findings, we propose that the dualistic nature of *cis*–*trans* isomerization of proline residues restricts the yield of properly folded protein from the total amount of denatured protein to be inversely proportional to two to the power of the number of prolines in the sequence (∼1/2*^n^*, where *n* is the number of prolines). In this regard, we accompanied our novel refolding protocol with an investigation into the effects of proline isomerization in the refolding of proteins. The structure of AID^153^ reveals the locations of four prolines, one of which is located on a flexible loop distal from the secondary and tertiary structures. This proline, Pro72, was chosen as the site for a point mutation to a neutrally charged asparagine (P72N; mAID^153^). Parallel experiments were conducted utilizing AID^153^ and mAID^153^ to reveal a finding that reinforces the notion that prolines play a crucial role in protein folding, but challenges the widely believed notion that proline isomerization can be attributed to the slow phase in protein folding. Given how fruitful the AID^153^ model system has been in our investigations into proline, we proceeded to continue our exploration into one of the greatest mysteries of contemporary science: the general mechanism of protein folding.

The article "Hydrogen bonds are a primary driving force for de novo protein folding" was retracted in 2018. Reasons: contaminated materials; errors in the data; errors in the results or conclusions.

How proteins fold has remained a topic of intense research efforts for more than half a century. Indeed, this topic was deemed to be one of the 125 most compelling questions faced by scientists (Kennedy, 2005 ▸). Despite reports detailing several significant milestones during the last few decades, how proteins transition from a completely unfolded state to their native structure is still not well understood. In the mid-1960s, a group of scientists produced the first case of a synthetic active protein: bovine insulin (Tsou, 1995 ▸; Niu *et al.*, 1964 ▸; Du *et al.*, 1961 ▸; Wang *et al.*, 1965 ▸). Subsequent studies subjected various proteins, including ribonuclease A (RNase A), to refolding experiments to show that primary protein sequences determine tertiary protein structures (Anfinsen, 1973 ▸; Anfinsen & Haber, 1961 ▸; Haber & Anfinsen, 1961 ▸, 1962 ▸). Others have speculated that certain aspects of the RNase A secondary structure may have persisted under the denaturing conditions used in these initial experiments (8 *M* urea for 4.5 h). More recent research revealed that proteins subjected to similar denaturing conditions were mostly denatured, but not completely unfolded; the denatured proteins were structurally heterogeneous, yet retained some native-like structures (Chang, 2009 ▸). Moreover, the degree of conformational heterogeneity among the denatured proteins significantly impacted on how protein folding occurred (Chang, 2009 ▸). Efforts to synthesize active RNase A (Gutte & Merrifield, 1971 ▸; Hirschmann *et al.*, 1969 ▸) and insulin have reinforced the theory that the primary protein sequence does completely determine the final tertiary structure. Insulin, for example, is composed of two small peptides: a 21-residue subunit A and a 30-residue subunit B. Each subunit contains a single disulfide bridge, and the two subunits are held together by a third inter-subunit sulfur–sulfur bond (Tsou, 1995 ▸; Niu *et al.*, 1964 ▸; Du *et al.*, 1961 ▸; Wang *et al.*, 1965 ▸). Despite the protein being small, *de novo* folding of insulin has been proven to be complicated, yet achievable. Since these initial experiments, numerous small proteins have been synthesized and folded into their native forms *in vitro*. For instance, smaller peptides have been subjected to stepwise covalent ligation to construct larger proteins, such as human immunodeficiency virus (HIV) protease (Muir & Kent, 1993 ▸; Torbeev & Kent, 2007 ▸; Kent, 2009 ▸) and the membrane potassium channel KcsA (Valiyaveetil *et al.*, 2002 ▸). These successful examples, however, were all relatively small targets (<130 residues). Of note, the folding process for each individual protein was different, and no common themes have emerged. Success with membrane proteins is particularly rare (Booth & Curnow, 2009 ▸; Miller *et al.*, 2009 ▸). Moreover, the recovery rate of the starting material is fairly low; for example, only approximately 1% of synthesized insulin peptides were recovered as completely folded protein (Tsou, 1995 ▸; Niu *et al.*, 1964 ▸; Du *et al.*, 1961 ▸; Wang *et al.*, 1965 ▸). Additionally, recent computer-modeling techniques that have attempted to predict protein folding have not uncovered any general folding principles (Portman, 2010 ▸; Dill *et al.*, 2008 ▸; Das & Baker, 2008 ▸). Over the past two decades, we have carried out thousands of protein-folding and unfolding experiments to explore the underlying mechanisms. In a previous study, we revealed that more than 100 urea molecules bind to protein only through hydrogen bonds at atomic-level resolutions. Combined with other biochemical and biophysical data, we concluded that protein denaturation by urea is caused by the disruption of protein main-chain hydrogen bonds (Wang *et al.*, 2014 ▸). Encouraged by this exciting discovery, we questioned whether *de novo* protein folding shares a similar trajectory. To our surprise, besides the critical dependence of protein folding on the number of proline residues, we found that proteins folded with greater efficacy at very high pH values (11.5–12.5). Further experiments revealed that peptide bonds are polarized at high pH values, which may in fact mimic the conditions of protein folding *in vivo*. Based on these novel discoveries, we concluded that hydrogen bonds are a primary driving force in *de novo* protein folding. In this regard, our study presents direct experimental observations that support a distinct theoretical protein-folding model.

The article "Hydrogen bonds are a primary driving force for de novo protein folding" was retracted in 2018. Reasons: contaminated materials; errors in the data; errors in the results or conclusions.

## 2. Materials and methods   

### 2.1. Protein expression and purification   

The DNA corresponding to the genes for wild-type (AID^153^) and P72N mutant (mAID^153^) activation-induced cytidine deaminase (AID) was cloned into a pET-28a vector containing an N-terminal His tag. AID^153^ and mAID^153^ were expressed in *Escherichia coli* BL21(DE3) cells. The cell cultures were grown to an *A*_600_ of about 1.0 and were induced with a final concentration of 1.0 m*M* isopropyl β-d-1-thio­galactopyranoside for 4 h at 37°C. The cells were resuspended in nickel-binding buffer (50 m*M* Tris–HCl pH 8.0, 1 *M* NaCl, 1 m*M* PMSF) and lysed using a sonicator (Fisher Scientific Sonic Dismembrator Model 500) at 35% power, 10 s on, 5 s off for 20 min. The lysate was centrifuged at 16 000 rev min^−1^ and 4°C for 30 min. The supernatant was discarded and the pellet was resuspended in 9 *M* urea. Upon homogenization, the inclusion-body solubilized lysate was pre-chilled on ice and sonicated at 100% for 2 min. The solution was loaded onto 10 ml Ni–NTA resin (GE Healthcare), washed with 9 *M* urea and eluted with buffer consisting of 9 *M* urea, 1 *M* imidazole. The eluted product was placed in a 6000–8000 molecular-weight cutoff (MWCO) dialysis membrane (Spectrum Laboratories Inc.) and submerged in 1 l refolding buffer *A* (50 m*M* Tris–HCl pH 8.0, 1 *M* NaCl, 4 *M* urea, 15 m*M* β-mercaptoethanol, 1 m*M* PMSF) at 4°C for 12–16 h. The buffer was replaced with 1 l refolding buffer *B* (50 m*M* Tris–HCl pH 8.0, 1 *M* NaCl, 3 *M* urea, 15 m*M* β-mercaptoethanol, 1 m*M* PMSF) and incubated at 4°C for 8–12 h. The buffer was replaced with 1 l refolding buffer *C* (50 m*M* Tris–HCl pH 8.0, 1 *M* NaCl, 2 *M* urea, 15 m*M* β-mercaptoethanol, 1 m*M* PMSF) and incubated at 4°C for 12–16 h. The contents of the dialysis membrane were loaded onto 5 ml Ni–NTA resin, washed with nickel-binding buffer and eluted with nickel-binding buffer containing 500 m*M* imidazole. The eluted product was concentrated and purified on a Superdex 200 10/300 GL column (GE Healthcare) previously equilibrated with nickel-binding buffer containing 15 m*M* β-mercaptoethanol.

### 2.2. Protein crystallization and data collection   

Purified AID^153^ was concentrated to 20 mg ml^−1^. The crystals were grown at 4°C by sitting-drop vapor diffusion against a reservoir consisting of 4 *M* potassium formate, 0.1 *M* bis-tris propane pH 9.0, 2%(*w*/*v*) PEG monomethyl ether 2000. The crystals were briefly soaked in the crystallization solution supplemented with 20% glycerol and flash-cooled in liquid nitrogen. X-ray diffraction data were collected at the Advanced Photon Source (APS) at Argonne National Laboratory. The data were indexed, integrated and scaled using the *HKL*-2000 program suite. Five separate data sets were merged and used for structure determination. Purified DapA and refolded DapA were crystallized *via* sitting-drop vapor diffusion against a reservoir containing 2 *M* K_2_HPO_4_ pH 9.8.

The article "Hydrogen bonds are a primary driving force for de novo protein folding" was retracted in 2018. Reasons: contaminated materials; errors in the data; errors in the results or conclusions.

### 2.3. Structure determination and refinement   

The AID^153^ structures were determined by molecular replacement using *phenix.automr* with the structure of a variant human AID (PDB entry 5jj4; Pham *et al.*, 2016 ▸) as a template. Iterative rounds of model rebuilding and simulated-annealing torsion-angle refinement were performed using *Coot* and *REFMAC*5. The data-collection and structure-refinement statistics are shown in Table 1 ▸. Atomic coordinates and structure factors have been deposited in the Protein Data Bank under accession code 5w09.

### 2.4. Refolding experiments followed by Bradford assay   

Following the isolation of 9 *M* urea-solubilized AID^153^ and mAID^153^ and prior to refolding, the samples were loaded into a glass flask and boiled for 15 min. The boiled samples were cooled to room temperature, the concentration of the protein was measured, and the refolding and purification method outlined above was followed. From the Superdex 200 10/300 GL column, fractions collected corresponding to the soluble form of AID^153^ used for crystallization were compared with fractions collected corresponding to the entirety of the non­soluble form of AID^153^. The protein concentrations of these two fractions was measured *via* the Bradford assay and a ratio was determined. This ratio was used to extrapolate the concentration of soluble AID^153^ that was present in the Ni–NTA-eluted product prior to injection into the Superdex 200 10/300 GL column. This value was used to assess the difference in concentration between AID^153^ and mAID^153^.

### 2.5. Refolding protein at various pH values   

Separately, purified ribulose bisphosphate carboxylase large chain (RuBisCo), dihydrodipicolinate synthase (DapA), 5,10-methylenetetrahydrofolate reductase (METF) and 5,10-methylenetetrahydrofolate reductase (METK) were subjected to unfolding (10 *M* urea, 50 m*M* Tris–HCl pH 8.0, 15 m*M* β-mercaptoethanol) for 1 h at room temperature. The unfolded protein was concentrated to a final volume of 1 ml (1 mg ml^−1^). The unfolded protein was titrated into 100 ml buffer at varying pH values. The buffer recipes for a pH range of 8.5–13 are listed in Supplementary Table S1. The refolded proteins were concentrated and subjected to a Superdex 200 10/300 GL column (GE Healthcare) for comparison with the native protein.

### 2.6. Fast protein refolding   

Following the inclusion-body purification steps and prior to refolding, as outlined above, the Ni–NTA-eluted products containing AID^153^ or mAID^153^ solubilized in 9 *M* urea were boiled to a completely denatured state and cooled to 22°C; NaCl was added to a final concentration of 1 *M* and the pH was adjusted to a value of 11.5. This solution was placed in a 6000–8000 MWCO dialysis membrane (Spectrum Laboratories Inc.) and submerged in 1 l refolding buffer *D* (200 m*M* Tris–HCl pH 8.0, 1 *M* NaCl, 15 m*M* β-mercaptoethanol, 1 m*M* PMSF) at 22°C for 4 h. The contents of the dialysis membrane were loaded onto 5 ml Ni–NTA resin, washed with nickel-binding buffer and eluted with nickel-binding buffer containing 500 m*M* imidazole. The concentration of the soluble fraction of well folded AID^153^ or mAID^153^ in the total elution was evaluated following the procedure outlined above.

The article "Hydrogen bonds are a primary driving force for de novo protein folding" was retracted in 2018. Reasons: contaminated materials; errors in the data; errors in the results or conclusions.

### 2.7. Small-angle X-ray scattering (SAXS)   

Native protein samples in buffer at pH 8.5 and refolded samples in buffers at various pH values were adjusted to concentrations of 1.0, 2.0, 4.0 and 5.0 mg ml^−1^ for SAXS experiments. SAXS data were collected on ALS beamline 12.3.1 at Lawrence Berkeley National Laboratory, Berkeley, California, USA (Hura *et al.*, 2009 ▸). Incident X-rays were tuned to a wavelength of 1.0 Å at a sample-to-detector distance of 1.5 m, resulting in scattering vectors (*q*) ranging from 0.001 to 0.32 Å^−1^. The scattering vector is defined as *q* = 4πsinθ/λ, where 2θ is the scattering angle. All experiments were performed at 20°C, and the data were processed as described previously (Hura *et al.*, 2009 ▸). Briefly, the data were acquired at short and long time exposures (0.5 and 5 s, respectively), and were then scaled and merged for calculations using the entire scattering profile. *FoXS* (Schneidman-Duhovny *et al.*, 2010 ▸) was used to compute the theoretical scattering profiles and accurately fit the experimental data.

### 2.8. Ultraviolet resonance Raman (UVRR)   

All UVRR spectra were collected on a custom-built UVRR spectrometer, which was designed based on previously published studies (Balakrishnan *et al.*, 2008 ▸; Lednev *et al.*, 2005 ▸). A tunable, frequency-quadrupled, titanium–sapphire laser (Coherent, Santa Clara, California, USA), pumped by the second harmonic of an Nd:YLF laser, was used as the excitation source. The sample was circulated using a gear pump (model 75211-10; Cole Parmer, Vernon Hills, Illinois, USA) through a temperature-controlled sample chamber and water-jacketed reservoir maintained at ∼7°C; this apparatus was designed in-house and was manufactured by Mid Rivers Glassblowing, Saint Charles, Missouri, USA. A thin film of the sample was created by passing the solution through a 19-gauge needle and between two thin Nitinol wires (0.005 mm in diameter; Small Parts, Miramar, Florida, USA). The sample film was directly irradiated by the incident excitation beam. A continuous stream of nitrogen gas was used to eliminate ambient oxygen from the sample chamber. The excitation wavelength was 197 nm. Raman scattering was collected over 135° of backscattering geometry and dispersed using a 1.25 m spectrometer (Horiba Jobin Yvon, Edison, New Jersey, USA) equipped with a 3600 groove mm^−1^ grating. The spectrometer was equipped with a back-illuminated, phosphor-coated, liquid-nitrogen-cooled Symphony CCD camera (Horiba Jobin Yvon, Edison, New Jersey, USA) with a chip size of 2048 × 512. The laser power at the sample chamber was kept below 0.5 mW to avoid sample degradation (Wu *et al.*, 2003 ▸). Each spectrum was collected over 150 min, which resulted in 60 individual spectra. The spectra were collected and exported in CSV format using the *Synergy* software (Horiba Jobin Yvon, Edison, New Jersey, USA). The spectrum of cyclohexane and the peak positions reported in Ferraro & Nakamoto (1994 ▸) were used to calibrate the UVRR spectra. The UVRR spectra were analyzed using *MATLAB* v.7.1 (Mathworks, Natick, Massachusetts, USA). The spectra were averaged and cosmic rays were removed using a program that was written in-house. Nonlinear least squares was then used to fit the spectra to a series of mixed Gaussian and Lorentzian bands, a process that was performed using a program that was written in-house for the *MATLAB* environment to approximate results obtained with the computationally intensive Voigt line shape.

The article "Hydrogen bonds are a primary driving force for de novo protein folding" was retracted in 2018. Reasons: contaminated materials; errors in the data; errors in the results or conclusions.

## 3. Results and discussion   

### 3.1. Overall crystal structure of AID^153^   

Heterologous protein expression of a pET-28a vector containing a full-length AID insert with an N-terminal His_6_ tag yielded protein that was homogenously truncated at the Glu153 position (Supplementary Fig. S1) exclusively in the inclusion bodies. The protein was purified utilizing a novel gradational refolding technique (see §[Sec sec2]2) and crystallized in space group *P*2_1_. Phases were determined by molecular replacement using the structure of the human AID variant AIDv(Δ15) (Pham *et al.*, 2017 ▸) as a search model. The crystal was shown to exhibit pseudo-merohedral twinning. High-resolution data were collected at APS to 2.0 Å resolution. Five separate data sets were merged and the structure was subjected to refinement in *REFMAC*5 using two twin operators simultaneously: (*l*, *k*, −*h* − *l*) and (−*h* − *l*, *k*, *h*). Refinement statistics are shown in Table 1 ▸.

The AID^153^ monomer exhibits the canonical APOBEC fold with an α–β–α supersecondary-structural element, comprised of five α-helices enveloping the inner five-stranded β-sheets, that forms the core catalytic site of a cytidine deaminase (CDA) domain (Figs. 1*a* and 1*b* ▸). The missing residues 154–198 are predicted to form the last α6 helix. A previously reported APOBEC3G dimerization model suggests the involvement of the α6 helix in the head-to-tail dimer conformation, resulting in a continuous DNA-binding groove (Lu *et al.*, 2015 ▸). Given the curiously homogenous truncation before the α6 helix resulting in AID^153^, despite the induction of an expression plasmid containing full-length AID, the inability to isolate soluble full-length AID may stem from the cellular instability that results from high-order oligomerization of full-length AID utilizing the α6 helix (Fig. 1*c* ▸). Interestingly, AID^153^ shows a single peak on a gel-filtration column with the molecular weight of an AID^153^ dimer, indicating the possibility of alternative dimerization mechanism(s), such as head-to-head or tail-to-tail, rather than the reported head-to-tail APO3G model exclusively (Shandilya *et al.*, 2010 ▸). The question of the cellular mechanism that leads to disruption of oligomerization, uniform truncation after the Glu153 site and inclusion-body trafficking remains to be answered.

The article "Hydrogen bonds are a primary driving force for de novo protein folding" was retracted in 2018. Reasons: contaminated materials; errors in the data; errors in the results or conclusions.

Structural similarity searches performed using the *DALI* server with AID^153^ as the query revealed similarity to members of the APOBEC family. The structures of AID^153^ and 146 aligned residues of AIDv(Δ15) (PDB entry 5jj4) superimposed with a root-mean-square deviation (r.m.s.d.) of 1.5 Å and a *Z*-score of 19.0. The structures of AID^153^ and over 145 aligned residues of numerous APOBEC3G structures (PDB entries 3v4j, 3v4k, 3ir2, 3e1u, 3iqs, 4rov and 4row) superimposed with an r.m.s.d. in the range 1.9–2.1 Å and a *Z*-score in the range 17.0–18.0. High structural similarity with an r.m.s.d. of <2.5 Å and a *Z*-score of >15.0 was also revealed between AID^153^ and APO3B, APO3A, APO3F and APO3C. The structure of AID^153^ appears to exhibit similarities, in terms of the overall fold, to previously reported structures of APOBEC family members.

### 3.2. Differences between crystal structures   

The previously reported crystal structure of AIDv(Δ15) contains numerous mutations at the N-terminus in the sequences responsible for forming the α1 helix and β1 sheet. Upon comparison with the structure of AID^153^, the impact of these numerous mutations is revealed. The most significant difference in structure compared with AID^153^, which contains all wild-type residues up to the Glu153 truncation site, is the presence of a continuous β2 sheet in AIDv(Δ15) and of a discontinuous β2/β2′ sheet containing a short bulging loop (termed the β2-bulge) in AID^153^ (Fig. 2 ▸ *a*). The resulting β2-bulge-β2′ topology is a feature that is present in APO3A, the APO3G C-terminal CDA domain and the APO3B C-terminal CDA domain, whereas the feature is not present in the Z2-type structures of APO3C, the APO3F C-terminal CDA domain, the APO3G N-terminal CDA domain or in APO2 (Salter *et al.*, 2016 ▸). Although the exact function of the bulge is unclear, it is suggested that the β2 strand interacts with the adjacent CDA domain in a bulge-dependent manner, or may possibly play a role in the quaternary organization of single-domain APOBEC family member proteins such as APO3A. This bulge is an intrinsic feature among some APOBEC family members, and the structure of AID^153^ reveals the novel finding that may categorize AID as a member of the β2-bulge-containing APOBEC family. Furthermore, in the instance where the bulge indeed plays a role in quaternary organization and/or higher order oligomerization as proposed, this may explain why Pham and coworkers were able to obtain soluble AIDv(Δ15), which lacks the presence of the β2-bulge.

The article "Hydrogen bonds are a primary driving force for de novo protein folding" was retracted in 2018. Reasons: contaminated materials; errors in the data; errors in the results or conclusions.

In AID, the CDA domain consists of three zinc-coordinating residues (His56, Cys87 and Cys90) and a proton-shuttle residue (Glu58). The AID^153^ structure presented in our study was solved in the absence of zinc. Interestingly, when compared with the CDA motif of the zinc-bound AIDv(Δ15), the orientation of Glu58 appears significantly different. In the presence of zinc, Glu58 is oriented towards the active site, as well as interacting with a water molecule coordinating to the zinc ion. In the absence of zinc, Glu58 is oriented away from the active site and the water molecule is absent. A minor, yet noticeable, difference can also be seen for the His56 residue, where the imidazole ring appears to be rotated by ∼60° in the zinc-free AID^153^ compared with the His56 bound to zinc in the AIDv(Δ15) structure (Fig. 2 ▸ *b*). Shaban and coworkers reported the structure of zinc-free APOBEC3F and revealed the formation of a disulfide bond between the cysteines that would otherwise coordinate zinc in their reduced form (Shaban *et al.*, 2016 ▸). AID^153^ exhibited no such disulfide-bond formation. Despite the difference in the active-site residue conformation, our results demonstrate that maintenance of the overall structural integrity of AID^153^ does not require zinc. Furthermore, the coherent orientation of Glu58 away from the active site in the absence of zinc may suggest that metal coordination is a strategy for regulating the activity of AID.

### 3.3. The number of proline residues determine the final refolding yield   

As described below, we have developed a novel refolding procedure for AID^153^ that could be applied to other proteins. Following the refolding and Ni–NTA purification process of AID^153^, 16.6 ± 1.70% of the total inclusion-body solubilized and isolated AID^153^ was in the native form, which shows a single peak on a gel-filtration column (Supplementary Fig. S2*a*). This peak was used for crystallization and yielded the crystals used for the final structural determination. After collecting the improperly folded and aggregated AID^153^ portion contained in the Ni–NTA flowthrough, we resolubilized the content in 9 *M* urea and conducted a second run of refolding and purification, resulting in a final yield of 5.30 ± 2.18%. The unfolded AID^153^ was subjected to a third run, resulting in the recovery of only 3.33 ± 2.6% of native AID^153^ (Fig. 3 ▸ *b*). To account for the decrease in recovery yield in each subsequent refolding and purification trial, we hypothesized that proline residues are the major determinants of protein refolding. The rationale for this hypothesis was inspired by the numerous protein-folding experiments that we have performed in past decades, in which we observed an interesting phenomenon. When purified proteins were subjected to denaturation for a short period of time (∼1 h, 10 *M* urea, room temperature) we were able to recover over 90% of well folded protein when high-pH refolding procedures were applied, as expounded upon below. However, when the purified proteins were subjected to denaturation for a prolonged period of time (>16 h, 10 *M* urea, room temperature) virtually no refolded protein could be recovered. Although we hypothe­sized that proline isomerization was the mechanism behind this disparity in the recovery yield, the protein candidates that we experimented with (RuBisCo, DapA, METF, METK *etc.*) contained too many essential proline residues to meaningfully test our hypothesis. Fortuitously, AID^153^ contains only four proline residues, which made this protein an ideal model to test our long-anticipated hypothesis.

The article "Hydrogen bonds are a primary driving force for de novo protein folding" was retracted in 2018. Reasons: contaminated materials; errors in the data; errors in the results or conclusions.

The role of proline in the process of protein refolding has been widely studied. Most results propose that the isomerization of proline residues leads to a slow refolding process in which the energy generated from correct protein folding overcomes the improper proline configuration. According to the final structure of AID^153^, all four proline residues are present in the *trans* form (Fig. 3 ▸ *a*). We reason that crude inclusion bodies may contain a higher percentage of the *trans* form of AID^153^ compared with the completely denatured form, since all amino acids, including proline, are translated in the *trans* form from ribosomes. Otherwise, an elegant report showed that short peptides with a proline residue coupled to any other residue, on average, generate almost equal amounts of the *cis* and *trans* forms of proline in the peptides (Zoldák *et al.*, 2009 ▸). In the context of our experiment above, when the Ni–NTA flowthrough is resolubilized in 9 *M* urea, unfolded protein molecules with the correct proline configurations are provided with another opportunity to fold properly, as well as allowing some minute population of unfolded protein molecules with incorrect proline configurations to adopt the correct proline configurations and proceed to fold properly. Our data suggest that each subsequent trial of resolubilizing the flowthrough reduces the relative amount of unfolded proteins with the correct proline configurations, as well as demonstrating that unfolded proteins with incorrect proline configurations yield little to no well folded proteins, owing to statistical improbability given that AID^153^ contains four prolines.

### 3.4. A point mutation of a proline residue to an asparagine led to a doubled yield of completely denatured AID^153^   

We hypothesized that if we completely denature AID^153^, the final yield of refolded protein should remain a constant value. Moreover, if we assume that all four proline residues have an equal probability of *cis* and *trans* configurations, while only four *trans* configurations corresponding to the ‘correct’ set could yield native-form AID^153^, the theoretical final yield should be (1/2^4^) × 100% = 6.25%. Our results appear to corroborate our hypothesis. AID^153^ dissolved in 9 *M* urea at pH 9.0 was boiled at 100°C for 15 min in order to ensure that no secondary structure was present and that there was an entirely random distribution of proline isomers in the AID^153^ solution. Starting from this completely denatured AID^153^, the final yield of refolded native AID^153^ was 3.45 ± 0.67% (Fig. 3 ▸ *b*). Accounting for experimental errors, our observed value of 3.45 ± 0.67% appears to be consistent with the expected theoretical value of 6.25%. Notably, the enormous discrepancy in the yield of refolding boiled *versus* unboiled protein suggests that the slow phase of protein folding is unlikely to be owing to proline isomerization. The energy required to overcome the threshold of proline isomerization is too large to be achieved during the refolding process since the final free energy generated from protein folding (Kyte, 2007 ▸) is at a similar energy level to that of *cis* and *trans* isomerization of one proline residue (Eyles, 2001 ▸). This notion, in the context of protein folding, becomes more apparent when fathoming the energy barrier associated with multiple prolines in the incorrect configuration. To further confirm our proline-dependent hypothesis, we introduced a point mutation of Pro72 to asparagine (mAID^153^). In general, Asn is a preferred residue in turn or loop regions of proteins, similar to a proline residue, although proline is relatively much more rigid. To our satisfaction, one mutation of a Pro residue to Asn led to a nearly doubled yield of mAID^153^. A procedure to prepare completely denatured mAID^153^, identical to that of AID^153^, resulted in a final yield of 6.58 ± 0.75% (Fig. 3 ▸ *b*). When compared *via* gel-filtration chromatography and a thermal denaturation assay (Niesen *et al.*, 2007 ▸), the P72N mutation appears to have no distinguishable impact on mAID^153^ compared with AID^153^ (Supplementary Fig. S2). Taken to­gether, these data strongly support the conclusion that an incorrect proline configuration markedly impedes the folding of native AID^153^ and mAID^153^ from a completely unfolded state.

The article "Hydrogen bonds are a primary driving force for de novo protein folding" was retracted in 2018. Reasons: contaminated materials; errors in the data; errors in the results or conclusions.

### 3.5. Optimal condition for the refolding of AID^153^ at regular pH values   

A major bottleneck that needed to be overcome in the process of obtaining soluble AID^153^ was the protein-refolding process. Conventional protein-refolding strategies solubilize the inclusion body in a high concentration of a chaotropic agent, subject the blend to a chelating-affinity column and subsequently dilute or dialyze the eluate directly into a buffer containing a low concentration of a chaotropic agent or no chaotropic agent at all (Rudolph & Lilie, 1996 ▸). When variations of this method were applied in an attempt to refold AID^153^, the products contained noticeable precipitation and virtually no well folded protein was recovered. Our previous research revealed that the urea-driven disruption of hydrogen bonds is the main driving force in unfolding proteins (Wang *et al.*, 2014 ▸). The novel refolding strategy proposed in this study involves a slow, gradational reduction of urea. Numerous studies have shown that the inflection point between an unfolded and folded protein typically falls in the range 4–5 *M* urea at a pH of ∼8 (Klotz, 1996 ▸; Rodriguez-Larrea & Bayley, 2013 ▸; Song *et al.*, 2013 ▸). Under these conditions, the unfolded protein can participate in hydrogen bonds and ionic inter­actions as effectively as urea. These interactions can manifest differently, insofar as there is competition between inter­actions that favor secondary-structure formation *versus* interactions that favor unfolded aggregation and/or amyloid formation. In contrast to buffers containing a low concentration or an absence of urea, prolonged incubation (12–16 h at 4°C) of unfolded protein in 4–5 *M* urea permits aggregation and/or amyloid formation to be reversible and allows the protein to form more thermodynamically stable secondary structures prior to reducing the urea concentration any further. This novel refolding approach was crucial in allowing sufficient quantities of soluble natively folded AID^153^ to be purified and ultimately crystallized. However, as our understanding of the general protein-folding mechanism deepens, we have revealed that high pH can speed up the process drastically, as we describe below.

The article "Hydrogen bonds are a primary driving force for de novo protein folding" was retracted in 2018. Reasons: contaminated materials; errors in the data; errors in the results or conclusions.

### 3.6. Protein folding under high-pH conditions   

Although the slow, gradational reduction of urea in the refolding procedure described above is intended to minimize the unfolded aggregation of recombinant proteins extracted from inclusion bodies of *E. coli*, this lengthy *in vitro* refolding of AID^153^ does not accurately reflect *in vivo* protein-folding conditions. On the contrary, it is very well established that *in vivo* protein folding is relatively instantaneous (Kiefhaber, 1995 ▸; Torshin & Harrison, 2003 ▸). To address this temporal discrepancy between *in vitro* and *in vivo* protein folding, we sought to optimize the complete denaturation, refolding and purification assay of AID^153^ and mAID^153^ described above, with the intention of revealing insights into general protein-folding mechanisms. In our search to simulate a general *in vivo* protein-folding condition, we screened thousands of conditions using several protein candidates to discover that pH is a major determining factor as to whether or not an unfolded protein can be properly folded in the shortest time. Our results indicated that a pH range of 11.5–12.5 was optimal in re­covering protein. Specifically, we observed an explicit correlation between greater efficacy of protein folding and increasing pH. Among the protein candidates that we explored, this phenomenon was best demonstrated by several well characterized proteins: RuBisCo (Fig. 4 ▸ *a*), DapA (Supplementary Fig. S3*a*), METF (Supplementary Fig. S3*b*) and METK (Supplementary Fig. S3*c*). In the case of DapA, our proposed refolding procedure at high pH was efficient to the degree that we were able to obtain crystals of refolded DapA that appeared to be identical to the crystals obtained from native DapA under the same crystallization conditions (Fig. 4 ▸ *b*). To identify the mechanism behind the pH-dependent protein folding, we opted to use the well characterized protein DapA in a small-angle X-ray scattering (SAXS) experiment to evaluate the approximate shape of the protein in a pH-dependent manner. Consistent with our previous findings (Wang *et al.*, 2014 ▸), DapA appears to be completely unfolded at pH 12.5–13.0. Surprisingly, at pH 11.5–12.5 DapA appears to have a three-dimensional structure similar to that of the native form, whereas at pH 9.5 DapA is structurally identical to the native form (Fig. 4 ▸ *c*). The presence of native secondary structure at different pH values further confirmed this observation (Supplementary Fig. S4). These results suggest that proteins could fold into native forms at high pH values. Based on these findings, we proceeded to use post-boiled AID^153^ and mAID^153^ solubilized in a pH 11.5 and 9 *M* urea solution to perform a 4 h direct dialysis (not stepwise) against a buffer at pH 8.0 with no urea at room temperature. To our satisfaction, under these experimental conditions the final yield of refolded native AID^153^ was 2.09 ± 0.32% and the final yield of refolded native mAID^153^ was 3.52 ± 0.19% (Fig. 4 ▸ *d*). The overall yields of both AID^153^ and mAID^153^ are similar to the results derived from the protracted experiments at pH ∼8.0 described above. This simplified *in vitro* protein-refolding procedure starting at high pH values may better reflect the *in vivo* protein-folding process. Interestingly, Singh and coworkers reported a similar finding, in which their refolding protocol maximized the recovery yield from inclusion-body solubilized human growth hormone (hGH) at a pH of above 8.0, with an even greater yield of soluble protein being recovered as the pH increased to 12.5 (Singh & Panda, 2005 ▸).

The article "Hydrogen bonds are a primary driving force for de novo protein folding" was retracted in 2018. Reasons: contaminated materials; errors in the data; errors in the results or conclusions.

### 3.7. High pH induces main-chain polarization   

To explore the underlying mechanism of protein folding under high-pH conditions, we proceeded to examine the principal unit in the protein structure: the peptide bond. Peptide bonds are known to display resonance; this process makes the double bond between the C and O atoms and the single bond between the N and H atoms longer than average, whereas the single bond between the C and N atoms is shorter than average (Milner-White, 1997 ▸). We propose that at high pH, apart from resonance or conjugation, OH^−^ groups surrounding a completely unstructured or nascent peptide will induce a partial negative charge on the O atom and a partial positive charge on the C atom. At the same time, the OH^−^ groups will also affect the H atom from the amide, leading to a partial negative charge on the N atom and a partial positive charge on the H atom (Fig. 5 ▸ *a*). The exchange rate of the amide proton is known to increase dramatically at high pH values (>10; Bai *et al.*, 1993 ▸), while we revealed that the dissociation of protons on peptide amides occurs at a pH of ∼13 (actual; Wang *et al.*, 2014 ▸), although the theoretical p*K*_a_ value for the amide proton is close to 16.0 (Gilli *et al.*, 2009 ▸). Overall, high pH will lead to the formation of two electric dipoles. Interestingly, these types of dipoles have been described in native protein structures, and this feature, which has been confirmed by quantum-mechanics calculations, is widely used in modeling programs (Milner-White, 1997 ▸). Furthermore, recent studies showed that the carbonyl-amide groups from the side chains of glutamines/asparagines, acetylated lysines and/or a portion of NAD^+^ could play critical roles in some enzymatic reactions through the formation of an imidic acid intermediate (similar to the polarized peptide-bond structure shown above) under hydrophobic and negative charged environments both in the deacetylation process by the NAD-dependent deacetylase sirtuin-2 (SIRT2; Lee *et al.*, 2017 ▸; Wang *et al.*, 2017 ▸) and in hydrolases (Nakamura *et al.*, 2015 ▸).

The article "Hydrogen bonds are a primary driving force for de novo protein folding" was retracted in 2018. Reasons: contaminated materials; errors in the data; errors in the results or conclusions.

We hypothesized that during the protein-folding process the electric dipoles are stabilized and enhanced by hydrogen-bond formation within the protein. If this is the case, however, then why do these atoms fail to form hydrogen bonds to water molecules, which should also stabilize and enhance the electric dipoles, as suggested previously (Myshakina *et al.*, 2008 ▸)? We propose that the water molecules are steered away from the peptide backbone under high-pH conditions; this is similar to reversed-phase or hydrophobic interaction chromatography, in which hydrophobic surfaces appear at low or high pH levels (Dorsey & Cooper, 1994 ▸). To verify and confirm the potential electric dipoles under high-pH conditions, UV resonance Raman (UVRR) spectra were utilized. UVRR spectra can be used to detail conformational changes within protein main-chain backbones (Asher, 1988 ▸; Balakrishnan *et al.*, 2008 ▸; Lednev *et al.*, 2005 ▸). When proteins are excited at 190–220 nm, the stretching of individual bonds is represented by a specific peak in the spectrum. For example, primarily C=O double-bond stretching is detected at a wavenumber peak of ∼1650 cm^−1^ (amide I), whereas mixtures of N—H single-bond bending and C—N single-bond stretching are detected at wavenumber peaks of ∼1550 cm^−1^ (amide II) and ∼1300 cm^−1^ (amide III) (Asher, 1988 ▸; Balakrishnan *et al.*, 2008 ▸; Lednev *et al.*, 2005 ▸). UVRR spectra were obtained for an acetylated polyglycine peptide (Ac-GGGG) at four different pH levels: 3.0, 7.0, 10.0 and 12.0. As expected, the double bond between the C and O atoms was elongated at high pH levels, which was reflected by a decrease in the amide I wavenumber peak from 1661 to 1656 cm^−1^ from low- to high-pH conditions (Fig. 5 ▸ *b*). Although no significant changes were observed for amide II, a slight increase in the wavenumber peak representing amide III was detected, which may reflect a shortening of the C—N bond (Fig. 5 ▸ *b*). Because of interference from water molecules, bending of the N—H bond is difficult to identify within the spectrum. Nuclear magnetic resonance (NMR) experiments have already confirmed a rapid exchange rate of protons at high pH levels (Bai *et al.*, 1993 ▸; Udgaonkar & Baldwin, 1988 ▸). These results demonstrate that electric dipoles are created within peptide bonds under high-pH conditions. Because the electric dipoles are enhanced by hydrogen-bond formation within nascent peptide bonds in the absence of water, we can further deduce that hydrogen bonds are a primary force that drives protein folding.

The article "Hydrogen bonds are a primary driving force for de novo protein folding" was retracted in 2018. Reasons: contaminated materials; errors in the data; errors in the results or conclusions.

## 4. Concluding remarks   

This study reports the following five novel discoveries: the structure of AID^153^, the role of proline isomerization in protein folding, the general protein-folding procedure at high pH, the observation of native-like structures of proteins folded at higher pH values (up to 12.0) and the phenomenon of main-chain polarization at higher pH values (up to 12.0). These discoveries are within the context of greater discussions.

Despite the fundamental role that AID plays in antibody diversification, recombinant expression of this protein in *E. coli* or insect cells has been unfeasible owing to the propensity of the protein for aggregation. In our study, we report a twinned crystal structure of human AID exhibiting a homogenous truncation at the Glu153 site (AID^153^) at a resolution of 2.0 Å. Our structure reveals the novel finding that AID exhibits a β2-bulge, a topology that is featured in some members of the APOBEC family. In addition, our structure in the absence of zinc reveals a notably different orientation of the key catalytic residue Glu58 compared with zinc-bound AIDv(Δ15), which may be a metal-dependent regulatory mechanism to provide an additional level of complexity to prevent promiscuous mutations of nonspecific ssDNA targets. Unfortunately, our structure comes up short in addressing the true value of the long-awaited AID structure. Although all APOBEC family members share a conserved zinc-dependent deaminase motif within an α–β–α super-secondary-structural element, the variations in length, composition and spatial location of conserved secondary-structural features define the substrate specificity, quaternary structural organizations and protein–protein interactions. Owing to the truncation and twinning, which may explain the suboptimal data-collection and refinement statistics, our structure of AID^153^ may be no more than a placeholder until the full-length structure of AID is determined, which is expected to address the many mysteries surrounding AID from a structural standpoint. Nevertheless, given the difficulty in obtaining the native form of the AID protein in the field, the general protein-unfolding and refolding procedure derived from AID^153^ may be used as a universal protocol for many other proteins. Above all, given that solving a structure largely ensures the homogeneity of the protein and the reproducibility of a given procedure for obtaining the protein, the unique steps taken here in acquiring soluble AID^153^ provided us with a fortuitous opportunity to use this protein as a model to explore one of the most compelling questions in the field of life science: the underlying mechanism of protein folding.

The article "Hydrogen bonds are a primary driving force for de novo protein folding" was retracted in 2018. Reasons: contaminated materials; errors in the data; errors in the results or conclusions.

Given that ribosomes translate prolines in the *trans* configuration, the rate-limiting process of proline isomerization in protein folding may only be applicable to prolines that are *cis* in the native conformation of the protein. From an evolutionary standpoint, this stands to reason given that a specialized enzyme, prolyl isomerase, exists to overcome the enormous thermodynamic penalty associated with proline isomerization. Furthermore, studies show that there are severe impacts on the refolding kinetics of proteins that contain a native *cis*-proline when prepared in *in vitro* unfolding conditions that impel proline isomerization towards establishing the thermodynamically driven 1:4 *cis*:*trans* proline equilibrium levels. In this regard, Roderer *et al.* (2015 ▸) reported a dramatic acceleration in the refolding kinetics by more than four orders of magnitude, compared with the wild type, when a conserved *cis*-proline was mutated to alanine in thioredoxin. Interestingly, in the same report the mutation of the other four *trans*-prolines to alanine, while retaining the single *cis*-proline, resulted in a 27-fold slower refolding compared with the wild type. In another study by Osváth & Gruebele (2003 ▸), yeast phosphoglycerate kinase was shown to refold more rapidly when a single *cis*-proline was mutated to a histidine. Notably, this study suggests proline isomerization as an ‘additional’ slow phase, with another unaccounted-for source being the other reason behind the slow phase in protein folding; an observation that was also noted by Hacke *et al.* (2013 ▸). Skeptics of the contribution of proline to the slow phase, such as Dr Duncan Steel, offer alternative explanations as to the source of the slow phase that result from the disruption of incorrectly formed hydrogen bonds or unfavorable van der Waals contacts in the hydrophobic core of the protein, followed by reformation of the correct contacts (Subramaniam *et al.*, 1995 ▸). These findings are not mutually exclusive, and taken together may totally account for the slow phase in protein folding. In this regard, we found that proline residues, and most likely differences in the *cis* and *trans* configurations, are a key determinant of protein folding. An incorrect configuration of a given proline residue, which is unable to convert without the help of specific enzymes (for example prolyl isomerases) under *in vitro* refolding conditions, leads to an irreversible trap in protein folding. Starting from complete­ly unfolded proteins with the equilibrated probability distribution of *cis*- and *trans*-proline isomers, the final yield of properly folded protein will be close to the reciprocal of 2*^n^* (where *n* represents the number of prolines in the corresponding protein). Our study demonstrates this proposal using AID^153^ as a model. Further studies using other protein candidates containing a limited number of essential proline residues (less than five prolines, which are vital to the overall structure) is necessary in order to derive a general theory behind our proposed mechanism of the role of proline in protein folding. Interestingly, upon exposure to denaturing conditions for a prolonged period of time (>16 h), we failed to refold any native-form proteins from other protein candidates with a high number of proline residues, such as DapA, RuBisCo, METF and METK. This may be owing to the many random isoforms of proline residues among these proteins (data not shown). This could be indirect evidence to indicate the critical role of proline residues in the process of protein folding.

The article "Hydrogen bonds are a primary driving force for de novo protein folding" was retracted in 2018. Reasons: contaminated materials; errors in the data; errors in the results or conclusions.

In our previous report, we used NMR spectroscopy to show that protons from the amide moiety of Ac-GGGG start to dissociate at pH levels above 13.0, which was reflected by large chemical shifts in the neighboring CH_2_ groups (Wang *et al.*, 2014 ▸). On the other hand, a high occupancy of hydrogen on the amide was observed at pH 12.0 and lower, which was reflected by the small or nonexistent chemical shifts in the neighboring CH_2_ groups, although the exchange rate dramatically increased (Bai *et al.*, 1993 ▸). Those findings led us to propose that the denaturation of proteins at extremely high pH is driven by the disruption of main-chain hydrogen bonds, similar to protein denaturation by urea molecules (Wang *et al.*, 2014 ▸). Interestingly, in our current study we observed the initiation of protein folding at pH ∼12.0 or below through SAXS and circular-dichroism (CD) spectra (Fig. 4 ▸ *c*, Supplementary Fig. S3). Furthermore, we also observed a trend towards the polarization of main-chain amides using UVRR when the pH was increased to 12.0 (Fig. 5 ▸ *b*). Combined, these experimental data appear to demonstrate that pH 12.0 is a threshold for protein folding or unfolding. The sole pH dependence of protein folding and the dynamic status of main-chain amides at high pH values in our observed data require a proper interpretation of the underlying mechanism. In this regard, we propose that hydrogen bonds are a primary driving force for *de novo* protein folding.

The importance of hydrogen bonds as a primary driving force of protein folding is underappreciated largely owing to the contention of a widely accepted theory: the formation of hydrophobic cores as a primary driving force of protein folding. This underappreciation stems from the fact that protein-folding mechanisms are currently largely in the realm of theory, and experimental observations that support one theory or another are few and far between. The core of our reasoning starts with our empirical data, which demonstrate greater protein-folding efficacy at higher pH. The effects of hydrophobicity at higher pH is well understood and is the basis for common techniques such as reversed-phase or hydrophobic interaction chromatography during protein purification, where the targeted protein binds to hydrophobic resin when exposed to high-pH conditions (Dorsey & Cooper, 1994 ▸). The mechanism is understood to be owing to water molecules being steered away from the surface of unfolded proteins under alkaline conditions, which leads to a relatively anhygroscopic microenvironment surrounding the proteins (Dorsey & Cooper, 1994 ▸). We propose that owing to the reduction in the number of water molecules surrounding the protein, such an environment will weaken the contribution of the water surface tension to the hydrophobic effect during the protein-folding process, which may otherwise form nonspecific intramolecular hydrophobic interactions and lead to irreversibly misfolded proteins. As we outline below, overwhelming *in vivo* data support this hypothesis.

Here, our study provides observable evidence that alkaline conditions enhance the formation of secondary structures by preventing competing water molecules from forming hydrogen bonds to the peptide backbone and induce main-chain polarization to enhance secondary-structure formation. Interpretation of these directly observed data lead to the deduction of the potential general protein-folding mechanism *in vivo*. As reported, various trigger factors assist with folding as peptides exit the ribosome (Hartl & Hayer-Hartl, 2009 ▸; Kramer *et al.*, 2009 ▸; Kaiser *et al.*, 2006 ▸; Martinez-Hackert & Hendrickson, 2009 ▸; Wang & Tsou, 1998 ▸; Cabrita *et al.*, 2010 ▸). These trigger factors contain a functional domain with hydrophobic and negative charges on the surface (Hoffmann *et al.*, 2010 ▸). As the nascent peptide chain leaves the cramped ribosomal tunnel and is bound by a trigger factor, water molecules are excluded, the physical space limitation is removed and secondary structures begin to form automatically. Furthermore, the recurring theme of GroEL studies emphasizes three key points: (i) the closed chamber structure of GroEL decreases conformational entropy (Hayer-Hartl & Minton, 2006 ▸; Zhou & Dill, 2001 ▸; Betancourt & Thirumalai, 1999 ▸), (ii) there is an abundance of hydrophobic residues within the chamber (Sigler *et al.*, 1998 ▸; Xu *et al.*, 1997 ▸) and (iii) the binding of GroES leads to GroEL exposing numerous negatively charged side chains within the chamber (Tang *et al.*, 2006 ▸). Taken together, GroEL appears to have hallmark features that preclude nonspecific intramolecular hydrophobic interactions that may form irreversibly misfolded proteins if left situated in aqueous environments. These processes involving hydrophobic and negatively charged residues that are observed *in vivo* are analogous to protein folding driven by negative charges from OH^−^ under *in vitro* high-pH conditions. In both these *in vivo* and *in vitro* conditions, the ensuing anhygroscopic environment not only excludes the interference of water molecules from competing hydrogen-bond formation within the polypeptide main chain, but also disrupts the water surface tension to diminish entropy-driven hydrophobic effects to negligible levels. A negatively charged environment contributed by glutamic acids or aspartic acids could trigger the polarization of main-chain peptide bonds (or imidic acid formation), which will induce secondary-structure formation through the formation of main-chain hydrogen bonds and release free energy. When these factors are taken into account, we propose that hydrogen bonds are a primary driving force of *de novo* protein folding. Based on our current results and the reports of others, a comprehensive model of protein folding can be derived (Fig. 6 ▸).

The article "Hydrogen bonds are a primary driving force for de novo protein folding" was retracted in 2018. Reasons: contaminated materials; errors in the data; errors in the results or conclusions.

All evidence from both *in vitro* and *in vivo* data shown above indicates the critical roles of hydrophobic and negatively charged microenvironments. A key question that remains is: what roles do the side chains of amino acids play and how do they participate during the entire protein-folding process? In this regard, researchers have reported that driven by thermal stabilization, some amino acids prefer to form α-helices, some amino acids prefer to form β-sheets and some amino acids are secondary-structure disruptors (Chou & Fasman, 1974 ▸; Levitt, 1978 ▸; Malkov *et al.*, 2008 ▸; Minor & Kim, 1994 ▸; Pace & Scholtz, 1998 ▸). Furthermore, it was demonstrated by proton-accessibility experiments that some secondary structures form first, acting as a core, and others follow (Roder *et al.*, 1988 ▸). Based on these valuable observations, we propose that the side chains of amino acids are the determinants of secondary-structure forms (α-helix or β-sheet or random coil) after main-chain polarization both *in vivo* and *in vitro*. Taking these findings into account, our proposed scenario for the *de novo* protein-folding process is as follows: in a relatively hydrophobic and negative charged environment *in vivo* (for example a molecular chaperone) (i) polarization of the main chain induced by negative charge triggers secondary-structure formation (both α-helices and β-sheets), (ii) β-sheet pairing brings remote secondary structures together, (iii) hydrophobic side chains loosely group together within the quasi-aqueous chaperone chamber and (iv) upon re-exposure to the cytosol the clustering of hydrophobic side chains strengthen under the aqueous environment, ultimately establishing a set of hydrogen bonds that correspond to the native form of the protein.

In our previous report, we have demonstrated the following: (i) denaturation by urea is caused by the disruption of hydrogen bonds, (ii) the hydrophilic features of PEG could neutralize urea through hydrogen-bond competition and (iii) protein denaturation at high pH is triggered by the dissociation of protons on the main chain at pH 13.0 and above (Wang *et al.*, 2014 ▸). In this report, we demonstrate that (i) high pH values lead to the successful refolding of all protein candidates that we tested, (ii) secondary-structure formation is observable up to pH 12.0 by CD spectroscopy, (iii) partial native structure of a protein is detectable at pH 11.5–12.5 by SAXS and (iv) a positive trend towards main-chain polarization was observed as the pH increased to pH 12.0 by UVRR. Considering the sole dependence of protein folding and unfolding on the pH level, and with pH being the sole factor in determining the strength of hydrogen bonds within our *in vitro* protein-folding conditions, this transitive relation leads us to propose that hydrogen bonds are a dominant primary driving force of protein folding. Interestingly, studies into amyloidosis appear to vindicate our proposition. Amyloids, which are an exceptionally unique occurrence among misfolded proteins, are one of the strongest and stiffest structures and are formed exclusively by main-chain amides participating in intermolecular hydrogen bonds, whereas the side chains contribute nominally towards the overall shape (Qiang *et al.*, 2017 ▸; Lu *et al.*, 2013 ▸; Wasmer *et al.*, 2008 ▸; Fitzpatrick *et al.*, 2017 ▸). Given the pre-eminent role that amyloids play in numerous neurodegenerative disorders, the future of amyloid research may require the consideration of hydrogen bonds as a primary driving force in the formation of amyloids.

The article "Hydrogen bonds are a primary driving force for de novo protein folding" was retracted in 2018. Reasons: contaminated materials; errors in the data; errors in the results or conclusions.

## Supplementary Material

PDB reference: twinned human AID, 5w09

Supplementary Figures and Table.. DOI: 10.1107/S2059798317015303/qh5051sup1.pdf

## Figures and Tables

**Figure 1:** (*a*) Ribbon representation and electrostatic potential surface of the AID^153^ monomer. (*b*) Ribbon representation of AID^153^ (green) overlapped with the A3G (PDB entry 4rov; Lu *et al.*, 2015 ▸) head-to-tail dimer conformer (orange).

**Figure 2:** (*a*) Structural alignment of the β2 strands that exhibit a β2-bulge in AID^153^, the A3G C-terminus (PDB entry 3ir2; Shandilya *et al.*, 2010 ▸), the A3B C-terminus (PDB entry 5cqi; Shi *et al.*, 2015 ▸) and A3A (PDB entry 2m65; Byeon *et al.*, 2013 ▸) or its absence in A2 (PDB entry 2rpz; RIKEN Structural Genomics/Proteomics Initiative, unpublished work), A3C (PDB entry 3vow; Kitamura *et al.*, 2012 ▸), the A3G N-terminus (PDB 2mzz; Kouno *et al.*, 2015 ▸), A3F (PDB entry 4j4j; Siu *et al.*, 2013 ▸) and AIDv(Δ15) (PDB entry 5jj4; Pham *et al.*, 2016 ▸). (*b*) Alignment of the CDA domains, containing the key residues His56, Cys87, Cys90 and Glu58, of AID^153^ (green) and AIDv(Δ15) (beige). The magenta sphere represents a zinc ion and the red sphere represents a water molecule.

**Figure 3:** (*a*) Location of prolines in AID^153^. Pro72 was chosen as a site for point mutation to investigate the effects of proline in protein refolding. (*b*) 36–44 h protein-refolding procedure: the percentage of refolded protein concentration recovered relative to the 9 *M* urea-solubilized unfolded protein concentration. Subsequent runs of refolding and purifying AID^153^ from the Ni–NTA flowthrough results in decreased recovery. Upon complete denaturation *via* boiling, mAID^153^, which contains a point mutation at Pro72, led to the recovery of ∼91% more refolded protein compared with AID^153^.

**Figure 4:** (*a*) Size-exclusion chromatography assay of RuBisCo refolded at various pH values. When refolded at pH 7.5, RuBisCo predominantly formed misfolded aggregates that eluted at the void volume. As the refolding pH increased to 11.5, the resultant eluate better resembled the native protein. (*b*) Refolded DapA can be crystallized under the same conditions as used for native DapA. This demonstrates that the refolded protein has the same properties as the native protein. (*c*) Kratky plots of SAXS results for DapA refolding under different pH conditions. Three-dimensional structures of DapA were observed to begin formation at pH 12.5. (*d*) 4 h protein refolding procedure: the percentage of refolded protein concentration recovered relative to the 9 *M* urea-solubilized unfolded protein concentration. Upon complete denaturation *via* boiling, mAID^153^, which contains a point mutation at Pro72, led to the recovery of ∼68% more refolded protein compared with AID^153^.

The article "Hydrogen bonds are a primary driving force for de novo protein folding" was retracted in 2018. Reasons: contaminated materials; errors in the data; errors in the results or conclusions.

**Figure 5:** (*a*) Resonance at the amide under high-pH conditions leads to electric dipole formation. Electric dipole formation after the attack by OH^−^. (*b*) Resonance at the amide of Ac-GGGG under different pH conditions. The wavenumber representing amide I decreases from 1661 to 1656 cm^−1^ as the pH increases, reflecting elongation of the carbonyl double bond. The increase in the wavenumber peak of amide III from 1306 to 1309 cm^−1^ may reflect a shortening of the bond between the amide C and N atoms.

**Figure 6:** Proposed model for the folding of *de novo* proteins in a completely unstructured state.

**Table 1:** Summary of diffraction data and structure-refinement statistics Values in parentheses are for the highest resolution shell.

Data collection	
Wavelength (Å)	0.9795
Space group	*P*2_1_
Resolution (Å)	53.28–2.00 (2.051–1.999)
Unit-cell parameters	
*a* (Å)	61.458
*b* (Å)	28.359
*c* (Å)	61.512
Observed reflections	104857
Unique reflections [*I*/σ(*I*) > 0]	15662
Average multiplicity	6.7 (2.3)
Average *I*/σ(*I*)	23.6 (6.0)
Completeness (%)	99.91 (98.75)
*R*_merge_ † (%)	10.4 (42.7)
Refinement	
Resolution (Å)	53.28–2.00
Reflections [*F*_o_ ≥ 0σ(*F*_o_)]	
Working set/test set	12225/582
*R*_work_/*R*_free_ ‡ (%)	26.7/29.1
No. of protein atoms	1.453
No. of water atoms	151
Average *B* factors (Å^2^)	
All atoms	31.52
Protein	33.21
Water	19.70
Root-mean-square deviations	
Bond lengths (A)	0.016
Bond angles (°)	2.028
Ramachandran plot (%)	
Most favored regions	79.0
Allowed regions	19.0
Disallowed regions	2.0
Twin operators	(*l*, *k*, −*h* − *l*) and (−*h* − *l*, *k*, *h*)

† *R*_merge_ =  .

‡ *R* =   .
